# Epoetin alfa resistance in hemodialysis patients with chronic kidney disease: a longitudinal study

**DOI:** 10.1590/1414-431X20187288

**Published:** 2018-05-07

**Authors:** E.J.F. Santos, E.V. Hortegal, H.O. Serra, J.S. Lages, N. Salgado-Filho, A.M. dos Santos

**Affiliations:** 1 Hospital Universitário, Universidade Federal do Maranhão, São Luís, MA, Brasil; 2 Departamento de Saúde Pública, Universidade Federal do Maranhão, São Luís, MA, Brasil; 3 Programa de Pós-graduação em Ciências da Saúde, Universidade Federal do Maranhão, São Luís, MA, Brasil

**Keywords:** Epoetin alfa, Drug resistance, Renal insufficiency, Chronic disease, Renal dialysis

## Abstract

Anemia is an inevitable complication of hemodialysis, and the primary cause is erythropoietin deficiency. After diagnosis, treatment begins with an erythropoiesis-stimulating agent (ESA). However, some patients remain anemic even after receiving this medication. This study aimed to investigate the factors associated with resistance to recombinant human erythropoietin therapy with epoetin alfa (αEPO). We performed a prospective, longitudinal study of hemodialysis patients receiving treatment with αEPO at our reference hospital from July 2015 to June 2016. Clinical data was collected, and the response to αEPO treatment was evaluated using the erythropoietin resistance index (ERI). The ERI was defined as the weekly weight-adjusted αEPO dose (U/kg per week)/hemoglobin level (g/dL). A longitudinal linear regression model was fitted with random effects to verify the relationships between clinical and laboratory data and ERI. We enrolled 99 patients (average age, 45.7 (±17.6) years; male, 51.5%; 86.8% with hypertension). The ERI showed a significant positive association with serum ferritin and C-reactive protein, percentage interdialytic weight gain, and continuous usage of angiotensin receptor blocker (ARB) hypertension medication. The ERI was negatively associated with serum iron and albumin, age, urea reduction ratio, and body mass index. Our findings indicate that resistance to αEPO was related to a low serum iron reserve, an inflammatory state, poor nutritional status, and continuous usage of ARBs.

## Introduction

Anemia commonly complicates the last stage of chronic kidney disease (CKD) and is associated with increased morbidity and mortality and a decreased quality of life in dialysis patients (1,2). Several factors contribute to the development of anemia in patients with CKD, including nutritional deficiencies, an inflammatory state, and blood losses related to the dialysis procedure. However, the primary cause of anemia is erythropoietin (EPO) deficiency resulting from diminished production in the kidneys (3,4).

The correction of anemia in patients with CKD requires the use of erythropoiesis-stimulating agents (ESAs) such as epoetin alfa (αEPO). Intravenous iron therapy is used as an adjuvant to prevent iron deficiency and minimize the need for ESA (5,6). Nearly all hemodialysis patients worldwide take an ESA (7), and in Brazil, ESA is taken by an estimated 80% of dialysis patients (8). While anemia correction significantly improves patient quality of life and reduces mortality rates (2,9–11), the response of hemodialysis patients to ESA treatment varies, and hyporesponsiveness or resistance to ESA therapy occurs in 5–10% of patients with CKD (12,13 [Bibr B14]).

Iron deficiency is the primary cause of a poor response to ESAs. However, anemia persists in some hemodialysis patients even after adequate iron supplementation (13). Other causes of anemia include concomitant inflammation or infection, cancer, hemolysis, hemoglobinopathies, severe hyperparathyroidism, aluminum intoxication, vitamin B12 and folate deficiencies, inadequate dialysis, myelosuppressive agents, myelodysplasia, pure red cell aplasia, and thyroid dysfunction (9,12–17). Moreover, other clinical factors have been investigated including ESA and antihypertensive medication interactions, age, and body mass index (BMI) (18,19).

Patients that are hyporesponsive to ESAs have a higher risk of mortality from cardiovascular events and other causes (10,20,21) and must be identified. Further, it is necessary to determine which factors may limit the response to ESA treatment and optimize the management of anemia in chronic renal patients undergoing hemodialysis. Our main objective was to determine the factors associated with the resistance to αEPO treatment in patients receiving hemodialysis.

## Material and Methods

We conducted an analytical, longitudinal study of patients with CKD registered in the hemodialysis program of our reference hospital in the municipal district of São Luís, MA, Brazil, from July 2015 to June 2016. Patients (and replacements) were randomly selected by a raffle. All patients were ≥18 years of age and capable of communicating and had received ≥3 months of dialysis and treatment with αEPO at the time the study began. Our exclusion criteria included erythrocyte transfusion in the previous three months, significant acute or chronic bleeding, active malignant or hematologic disease, folate or vitamin B12 deficiency, thrombocytopenia, uncontrolled secondary hyperparathyroidism, clinical history of parathyroidectomy, clinical trial participation, major elective surgery, temporary dialysis access, and chronic hepatopathy.

The size of the sample was calculated based on the hemodialysis program population of 130 patients, an expected prevalence of ESA resistance of 25%, a 95% confidence level, and a 5% estimated error. The required sample (n=90) was increased by 10% to compensate for possible losses during data collection (n=99).

During their hemodialysis visit, the patients answered a structured questionnaire containing socioeconomic and demographic data (age, sex, skin color), and a clinical history was taken. The questionnaire was administered by trained interviewers. The skin color was self-reported and classified as white or non-white. The patient variables included comorbidities, medications, treatment time in hemodialysis, dry weight, percentage interdialytic weight gain, Kt/V index, and body mass index (BMI).

Blood samples were collected during the second hemodialysis session of the first week of each month, and hematological parameters were analyzed using an Advia 120 System (Siemens AG, Germany). Other parameters including the transferrin saturation (TSAT), ferritin level, alkaline phosphatase, parathyroid hormone, albumin, pre- and post-hemodialysis blood urea nitrogen, sodium, potassium, calcium, phosphorus, glutamate-pyruvate transaminase, glucose, creatinine, and ultra-sensitive C-reactive protein (CRP) were evaluated using a Cobas 6000 Analyzer with manufacturer reagents and controls (Roche Diagnostics, USA). Anemia was defined as hemoglobin <10.0 g/dL. The TSAT was calculated as the ratio of serum iron to total iron binding capacity.

The pre-hemodialysis weights at the first three sessions of each month were averaged and used to calculate the percent weight gain between two sessions of hemodialysis (%IDWG):

$$\%\text{IDWG=}\frac{(\text{average weight before dialysis}-\text{dry weight})\times 100}{\text{dry weight}}$$

The BMI was calculated as dry body weight/height^2^.

The Kt/V index was calculated using the Daugirdas equation as recommended by the National Kidney Foundation Disease Outcomes Quality Initiative (22):

$$\frac{Kt}{V}=-\ln(R-0.008\times t)+(4-3.5\times R)\;0.55\times \frac{UF}{V}$$

where *R* is pre-urea/post-urea, *t* is the duration of the session in hours, −ln the negative natural logarithm, *UF* the weight loss in kilograms, and *V* the anthropometric volume of distribution of urea in liters (0.55 x post-dialysis weight).

The erythropoietin resistance index (ERI) was defined as the weekly weight-adjusted αEPO dose (U/kg/week) divided by the hemoglobin level (g/dL) and calculated monthly to investigate resistance to αEPO treatment. We analyzed the ERI of all patients during the entire study period to calculate ERI quartiles and establish a resistance cut-off value. Patients in the upper quartile during the first trimester of the study were defined as ESA resistant in the baseline data.

Categorical variables are reported as percentages, and continuous variables as means±SD or medians (quartile 3 – quartile 1), according to the normality determined by the Shapiro-Wilk test.

The ERI variable was taken as the outcome of the longitudinal linear regression model with random effects. This model was utilized to investigate potential predictors of αEPO resistance. The independent variables included in the linear regression model referred to the sociodemographic, clinical, and laboratory data obtained. Independent variables with a P-value <0.2 in univariate analyses were selected for inclusion in the adjusted model, and only variables with a P-value<0.05 were independently associated with the outcome of the final model. Data were analyzed using STATA, version 14 (StataCorp LLC., USA).

The study was approved by the Research Ethics Committee of the University Hospital of the Universidade Federal do Maranhão (HUUFMA), and the participating patients were required to sign a consent form (Protocol 1.232.730/2015).

## Results

Of the 99 patients (mean age, 45.7 (±17.5); male 51.5%) that participated in this study, 87 remained until its completion. Cases were lost due to transplants, transfers, blood transfusions, and death. The median hemodialysis treatment length was 47 months. The hemodialysis prescriptions were similar concerning types of dialysis solution (acid concentrate and bicarbonate concentrate of 8.4%), dialysate flow (500 mL/min), dialyzer flux (low), frequency, and time of hemodialysis sessions (4 h three times a week). Only the blood flow was different among patients, with amplitudes between 300–400 mL/min.

Systemic arterial hypertension (SAH) was the most common cause of CKD (21.2%), followed by chronic nephropathy from a previous graft (20.2%), and diabetes mellitus (DM) (15.1%). SAH (86.8%), DM (26.2%), and cardiovascular disease (22.2%) were the most common comorbidities. Forty-four patients (44.4%) used an angiotensin receptor blocker (ARB) antihypertensive medication, and 36 (36.3%) received adjuvant intravenous iron (Table 1). When the study began, the Kt/V index mean was 1.5 (±0.3), the urea reduction ratio (URR) mean was 69.8±7.1, and the monthly average hemoglobin level was 10.2 g/dL (±1.7). The amplitude of variation of the average hemoglobin in the following year was 9.0–11.0 g/dL, and the prevalence of anemia varied between 24.1 and 51.1%.

**Table 1.** Baseline characteristics of the hemodialysis patients according to the epoetin alfa resistance in the first trimester of the study.

Variables	Resistant to Epoetin Alfa*		Total (n=99)	P-value
	No (n=78)	Yes (n=21)		
Age (years)	45 (57–31)	47 (61–36)	45 (58–31)	0.543^m^
Gender-female, n (%)	36 (45.5)	12 (60.0)	48 (48.4)	0.249^x^
HD vintage, months	46.5 (74–16)	49 (87–16)	47 (78–16)	0.989^m^
Body mass index, kg/m^2^	22.2 (26.2–19.8)	21.8 (23.4–20.2)	22.2 (25.5–19.8)	0.419^m^
Kt/V Index, %	1.5 (± 0.3)	1.5 (± 0.1)	1.5 (± 0.3)	0.495^t^
Arterial hypertension, yes (n, %)	68 (87.1)	18 (85.7)	86 (86.8)	1.000^x^
ARB use, yes (n, %)	33 (42.3)	11 (52.3)	44 (44.4)	0.211^x^
SHPT treatment, yes (n, %)	16 (20.2)	3 (15.0)	19 (19.1)	0.756^f^
Anemia, yes (n, %)	20 (25.6)	19 (90.4)	39 (39.3)	<0.001^x^
Urea reduction ratio, %	70.1 (± 7.1	68.5 (± 7.4)	69.8 (± 7.1)	0.391^t^
Interdialytic weight gain, %	3.6 (± 1.7)	3.5 (± 2.0)	3.6 (± 1.7)	0.769^t^
Red blood cells, n	4.1 x 106 (± 7.5 x 105)	3.4 x 106 (± 5.6 x105)	4.0 x 106 (± 7.8 x 105)	<0.001^t^
Hematocrit, %	34.8 (± 5.0)	26.8 (± 3.1)	33.1 (± 5.7)	<0.001^t^
Hemoglobin, g/dL	11.0 (± 1.5)	8.3 (± 0.9)	10.4 (± 1.8)	<0.001^t^
MCV, fL	83.8 (± 6.7)	79.3 (± 8.8)	82.8 (± 7.4)	0.010^t^
MCH, pg	26.6 (± 2.6)	24.6 (± 3.4)	26.2 (± 2.9)	0.006^t^
MCHC, g/dL	31.7 (± 0.98)	31.0 (± 1.61)	31.5 (± 1.17)	0.016^t^
Serum iron, µg/dL	53.5 (69–44)	54 (59–43)	54 (69–44)	0.709^m^
Ferritin, µg/L	509 (970.7–254)	546 (1006–231.8)	511 (994–245)	0.778^m^
TSAT, %	26 (32–20)	23 (30–18)	26 (32–20)	0.530^m^
PTH, pg/mL	287 (713–156)	475 (658–140)	313.1 (705.3–152.6)	0.955^m^
GPT, U/L	11 (14–7)	8 (11–7)	10 (13–7)	0.074^m^
Serum albumin, g/dL	4.1 (4.4–4.0)	3.9 (4.1–3.4)	4.1 (4.4–3.9)	0.006^m^
Glucose, mg/dL	111.5 (139–96)	119.0 (138–111)	115 (131–107)	0.335^m^
Serum phosphorus, mg/dL	5.1 (± 1.5)	4.8 (± 1.8)	5.0 (± 1.6)	0.496^t^
Serum calcium, mg/dL	8.8 (9.1–8.3)	8.7 (9.2–8.3)	8.8 (9.2–8.3)	0.744^m^
Serum sodium, mmol/L	139 (142–137)	138.5 (141–136)	139 (142–137)	0.319^m^
Serum potassium, mmol/L	5.4 (± 0.90)	5.0 (± 0.73)	5.3 (± 0.88)	0.685^t^
Serum creatinine, mg/dL	12.2 (13.9–8.3)	11.7 (14.0–8.8)	12.0 (14.0–8.8)	0.603^m^
CRP-US, mg/dL	0.3 (0.7–0.1)	1.1 (4.4–0.3)	0.4 (1.0–0.1)	0.005^m^
αEPO dose, UI/kg/week	131.6 (173.9–70.7)	222.2 (242.4–200)	161 (200–78)	<0.001^m^
ERI*, UI/kg/week/Hb	11.6 (17.5–5.7)	25.5 (29.5–19.5)	15.0 (21.9–6.4)	<0.001^m^

Monthly ERI ≥19.47 throughout the first trimester; ^t^independent samples *t-*test; ^m^Mann-Whitney test; ^x^chi-squared test; ^f^Fisher's exact test. Data are reported as means±SD or median (quartile 3 - quartile 1). HD: hemodialysis; Kt/V: quality of dialysis; ARB: angiotensin receptor blocker; SHPT: secondary hyperparathyroidism; MCV: mean corpuscular volume; MCH: mean corpuscular hemoglobin; MCHC: mean corpuscular hemoglobin concentration; TSAT: transferrin saturation; PTH: parathyroid hormone; GPT: glutamate-pyruvate transaminase; CRP-US: ultra-sensitive C-reactive protein; αEPO: epoetin alfa; ERI: erythropoietin resistance index.

All patients in this study were treated with the αEPO produced by Bio-Manguinhos/FIOCRUZ and it was administered subcutaneously after dialysis. αEPO resistance was present in all months of the study with a prevalence of 19.7–42.5%. The average ERI was 15.3 (±9.0) in the first month and ranged from 11.9 to 16.9 in the following months. Figure 1 shows the ERI values during the one-year study according to our baseline data analysis of ESA resistance.

**Figure 1.** Distribution of the monthly average erythropoietin resistance index (ERI) in hemodialysis patients with chronic kidney disease per the resistance to treatment with epoetin alfa in the baseline data. *Monthly ERI ≥19.47 throughout the first trimester.

Baseline patient characteristics according to αEPO resistance in the first trimester are presented in Table 1. We observed several expected associations with αEPO resistance including an increased prevalence of anemia, high median αEPO dose, and elevated ERI. We also observed that αEPO resistance was associated with the number of red blood cells, hematocrit, hemoglobin, mean corpuscular volume (MCV), mean corpuscular hemoglobin (MCH), mean corpuscular hemoglobin concentration (MCHC), serum albumin, and CRP.

The coefficients of the longitudinal linear regression model are shown in Table 2. In the non-adjusted regression model, we found that the ERI was negatively associated with age, URR %, BMI, serum iron, and serum albumin. The ERI was positively associated with SAH, %IDWG, ARB use, and CRP.

**Table 2.** Longitudinal linear regression model of the laboratory and clinical parameters associated with the erythropoietin resistance index in hemodialysis patients.

Variables	Non-Adjusted				Adjusted			
	*β*	95%CI		P-value	*β*	95%CI		P-value
Age (years)	−0.062	−0.088	−0.037	<0.001	−0.137	−0.174	−0.099	<0.001
Arterial hypertension, (yes *vs* no)	2.449	1.254	3.645	<0.001	−1.216	−3.377	0.954	0.270
Kt/V index, %	0.700	−0.260	1.660	0.153	11.61	−0.009	23.238	0.050
Urea reduction ratio, %	−0.089	−0.133	−0.045	<0.001	−0.380	−0.075	−0.004	0.047
Interdialytic weight gain, g	0.301	0.119	0.483	0.001	0.528	0.212	0.844	0.001
Body mass index, kg/m^2^	−0.390	−0.479	−0.302	<0.001	−0.211	−0.359	−0.624	0.005
ARB use (yes *vs* no)	3.919	3.102	4.737	<0.001	2.068	0.472	3.663	0.011
Serum iron, µg/dL	−0.092	−0.110	−0.074	<0.001	−0.094	−0.127	0.061	<0.001
Ferritin, µg/L	0.0007	−0.0005	0.002	0.164	0.001	0.0002	0.003	0.025
Serum albumin, µg/L	−6.990	−8.118	−5.862	<0.001	−1.816	−3.258	−0.375	0.013
Ultra-sensitive CRP, µg/L	0.238	0.083	0.393	0.003	0.119	0.057	0.181	<0.001

Kt/V: quality of dialysis; ARB: angiotensin receptor blocker; CRP: C-reactive protein; CI: confidence interval; ARB: angiotensin receptor blocker antihypertensive.

In the adjusted model, age, URR %, BMI, serum iron, and serum albumin were negatively associated with the ERI. ARB use, %IDWG, serum ferritin, and CRP were positively associated with the ERI (Table 2).

## Discussion

In this study, we evaluated the response to αEPO treatment using the weekly weight-adjusted dose of αEPO and hemoglobin level to calculate the ERI. Patient factors (age, URR, %IDWG, BMI), ARB use, and laboratory parameters (C-reactive protein and serum iron, ferritin, and albumin) were independently associated with αEPO resistance in chronic renal patients on hemodialysis in this 12-month study. Anemia was present in 24.4–51.1% of our patients throughout the study period. According to the Brazilian Society of Nephrology Chronic Dialysis Census, an estimated 26% of the 112,004 Brazilians receiving hemodialysis have hemoglobin <10 g/dL (8). However, this is a clinical condition that must be reversed, as a hemoglobin concentration <10 g/dL is associated with an increased prevalence of cardiovascular alterations, increased hospitalization ratio, decreased quality of life, and higher morbidity and mortality (1,2).

We treated anemic patients with αEPO and intravenous iron. While this regimen can increase hemoglobin levels to recommended values and decrease complications in hemodialysis patients (10,12), the treatment of anemia with an ESA can increase the risk of mortality; high dosages of the ESA and treatment resistance are the primary factors for this outcome (21,23,24). It is important to determine which factors limit the ability of αEPO to correct anemia in hemodialysis patients so that treatment can be optimized. We found some expected associations of first-trimester patient factors with treatment resistance that support the ERI's capacity to evaluate the αEPO treatment response. For example, the prevalence of anemia, the average dosage of αEPO, and the ERI were higher in treatment-resistant individuals. Furthermore, all red blood cell indices (number of red blood cells, hematocrit, hemoglobin, MCV, MCH, and MCHC) were lower in the patients resistant to αEPO.

We observed that age was negatively associated with the ERI. While it seems counterintuitive that older patients show a better response to αEPO treatment, similar results are consistently found in other studies evaluating hemodialysis patients (3,20,25 [Bibr B26]–27). We also observed a negative association between serum levels of albumin and the ERI, that is, an increase in albumin enhanced the response to αEPO. A positive association between the CRP level and the ERI was identified, that is, an increase in the CRP level resulted in increased resistance to treatment. We used CRP as inflammation marker, as it predicts resistance to ESA treatment (28). The positive association between the ERI and CRP values and index reduction with increased albumin are conditions that are classically described as limitations of anemia treatment with ESAs.

An increase in albumin may reflect the improvement of a hemodialysis patient's general state of health and is usually associated with decreased inflammation and oxidative stress, and an improved nutritional state (29 [Bibr B30]). Furthermore, some clinical conditions, such as malnutrition and inflammation, disrupt erythropoiesis and cause hypoalbuminemia (27,29–31). An evaluation of the inflammatory status is relevant to renal patients receiving chronic hemodialysis because the inflammatory state of CKD causes resistance to the medullary action of EPO (32). Our study supports this conclusion. The mechanism of this association might be post-inflammatory cytokines that, like interleukin and tumor necrosis factor, act on the erythropoietic progenitor cells, opposing EPO and stimulating apoptosis (32,33).

We also observed that an increased BMI was associated with an improved response to αEPO treatment. Previous studies demonstrated that ESA dose requirements and the ERI are inversely related to total adipose tissue in dialysis patients (19,34). The BMI is an important nutritional status marker in these patients. Unlike the general population, in hemodialysis patients, the overweight condition is associated with a better clinical prognosis (21); the lower the BMI, the larger the uremic toxin load (34).

We showed that the increased %IDWG was associated with a decreased response to αEPO. Excessive %IDWG is usually attributed to fluid and sodium overload. Abnormal thirst regulation, hormonal derangements, and social, cultural, and psychological habits may account for low compliance with fluid and salt restrictions. We observed the association between the ERI and %IDWG even after adjusting the regression model with variables of the nutritional status (albumin and BMI). We propose that the association occurs because of an increase of %IDWG might change body fluid status. If the patient is fluid-overloaded, he/she will have lower hemoglobin (35,36). However, further studies are necessary to analyze that association, because it is important to differentiate a high %IDWG resulting from high hydrosaline intake or from successful dietary intake.

Most patients were hypertensive (86.8%) and 44% were taking ARB class antihypertensive medication. We noted that ARBs were associated with a high ERI, and patients taking an ARB were more resistant to αEPO treatment. This type of antihypertensive medication interferes with the action of angiotensin II in various ways. Although the mechanism is not completely understood, ARBs might inhibit the αEPO liberation induced by angiotensin and elevate plasma levels of N-acetyl-seryl-aspartyl-lysyl-proline that impairs the recruitment of pluripotent hematopoietic cells (18,37).

The global management of hemodialysis patients includes iron reserve monitoring as an essential component, because iron deficiency is closely associated with an inadequate response to ESA treatment (6,38,39). Our results reflected this relationship and demonstrated that increased serum iron was associated with diminished treatment resistance. Serum ferritin, another marker of iron reserves, showed a positive association with αEPO resistance, and increased ferritin resulted in a diminished response to αEPO. The high prevalence of comorbidities in hemodialysis patients limits the use of ferritin as an iron deficiency parameter because it can be elevated in acute or chronic inflammation states and by malnutrition, all common conditions in this population (5). Inflammatory conditions, already established as an important factor limiting the response to ESA treatment in hemodialysis patients, are the probable cause of the positive association that exists between ferritin and the ERI (32,33).

The URR is a simple measure of urea reduction (%) during a hemodialysis session. In this study, an increased URR was accompanied by an improved response to the treatment of anemia with αEPO. A high URR may reflect an effective dialysis session, frequently related to an improved response to ESA treatment (13,15 [Bibr B16],^23^). However, the pre-dialysis urea concentration might be increased due to factors that are independent of the dialysis prescription, such as protein ingestion and protein catabolic rate. Thus, an increase in the URR might reflect an improvement in the patient's nutritional state (40), a factor that, as previously discussed, exerts an important influence on the response to anemia treatment with an ESA.

The management of anemia in hemodialysis patients is a clinical challenge because the etiology of anemia in patients with renal disease is multifactorial. One of the limitations of this study was not evaluating the direct contribution of food consumption on the %IDWG. However, our study population selection was designed to minimize the factors that directly affect anemia management, and we excluded patients with severe comorbidities, recent blood transfusion, and folate or B12 deficiencies. Thus, the consideration of the factors that we found to be associated with the ERI may facilitate the optimization of treatment for anemic hemodialysis patients, increasing the percentage of patients who achieve the recommended hemoglobin level and limiting the use of high-dose αEPO.

Our results demonstrated that age, URR, %IDWG, BMI, use of ARBs, and serum iron and albumin were independently associated with the ERI in hemodialysis patients. The prevalence of anemia and resistance to αEPO treatment were high in our study population. We verified that low serum iron reserve, an inflammatory state, poor nutritional status, and continuous use of ARBs limit the efficacy of αEPO treatment.
